# Pulmonary Embolism in COVID-19 Patients: A Retrospective Case-Control Study

This article has been retracted.

**DOI:** 10.7759/cureus.18887

**Published:** 2021-10-19

**Authors:** Fatimah A Alaithan, Mahdi H Aljawad, Asia H Ghawas, Abdulrahman S Althobaiti, Qusai A Almuslem, Mohammed H Bin Nasif, Faisal F Algharbi, Reem A Alshehri, Yousef K Al Gethami, Khaled W Altowayan, Fahad K Alzahrani, Amal A Suwaylih, Abdullah S Alwadai, Abdulmajeed M Badawi, Malak Alshammari

**Affiliations:** 1 Radiology, Dammam Medical Complex, Dammam, SAU; 2 Radiology, King Fahd University Hospital, Al-Khobar, SAU; 3 General Practice, Dhurma General Hospital, Dhurma, SAU; 4 General Practice, Al Faisaliah Primary Health Care Center, Dammam, SAU; 5 General Practice, Al Naeriyah Hospital, Dammam, SAU; 6 College of Medicine, King Saud University, Riyadh, SAU; 7 College of Medicine, King Khalid University Hospital, Riyadh, SAU; 8 College of Medicine, King Abdulaziz University, Jeddah, SAU; 9 College of Medicine, Taif University, Al-Taif, SAU; 10 College of Medicine, Hadhramout University, Al-Mukalla, YEM; 11 College of Medicine, King Khalid University, Abha, SAU; 12 College of Medicine, Imam Abdulrahman Bin Faisal University, Dammam, SAU

**Keywords:** pulmonary angiography, computed tomography, pulmonary embolism, hyper coagulopathy, covid-19

## Abstract

Background: Coagulopathy is a well-recognized complication in patients with coronavirus disease 2019 (COVID-19). Pulmonary embolism (PE) has substantial morbidity and mortality if the diagnosis is missed or the management is delayed. Computed tomography pulmonary angiography (CT-PA) is the imaging modality of choice for PE. Therefore, this study aimed to investigate the positive rate of CT-PA for PE among patients with COVID-19.

Methods: We conducted a retrospective study examining the diagnostic yield of CT-PA in patients with confirmed COVID-19 and compared it with that in patients without COVID-19. The study included all adult patients with confirmed COVID-19 who presented from June 2020 to June 2021.

Results: The study included 316 patients, including 158 patients with COVID-19, who underwent CT-PA for ruling out PE. Overall, 76 patients were found to have PE on the CT-PA scan, yielding a positive rate of 24.1%, with a significant difference between patients with COVID-19 (8.2%) and those without COVID-19 (39.9%). Further, 138 (87.3%) patients with COVID-19 had elevated D-dimer levels compared with 34 (21.5%) patients without COVID-19. A multivariable regression analysis model revealed that the smoking status (odds ratio [OR] = 1.94; 95% confidence interval [CI]: 1.4-3.8) and obesity (OR = 4.1; 95% CI: 1.5-8.9) were independent predictors of PE among patients with COVID-19. However, the elevated D-dimer level was not significantly associated with PE among patients with COVID-19 (OR = 0.7; 95% CI: 0.4-1.8).

Conclusion: The study found that the positive rate of CT-PA for PE was lower among patients with PE indicating probable overutilization of investigation in these patients. Additionally, patients with COVID-19 had a higher proportion of elevated D-dimer levels that may be a contributor to the increased investigation for PE. Lastly, patients with COVID-19 who were current smokers had a higher tendency of having PE.

## Introduction

Coronavirus disease 2019 (COVID-19) is caused by severe acute respiratory syndrome coronavirus 2 (SARS-CoV-2) that was first identified as the pathogen responsible for a cluster of pneumonia cases in Wuhan, China, at the end of 2019. It was officially declared as a pandemic by the World Health Organization on March 11, 2020 [1]. The diagnosis of COVID-19 is made by nucleic acid amplification using reverse-transcription polymerase chain reaction (RT-PCR) tests since its clinical features are non-specific. The most common presenting symptoms of COVID-19 include cough, fever, myalgia, headache, and dyspnea. While COVID-19 predominantly affects respiratory symptoms, the involvement of the organ systems is not uncommon [2]. Several studies highlighted the wide spectrum of complications seen in COVID-19, including cardiovascular, thromboembolic, neurologic, and inflammatory complications [3-5].

It became evident that patients with COVID-19 had a number of complex and varied coagulopathies predisposing them to a wide spectrum of thromboembolic conditions [6]. The pathogenesis of such coagulopathies is not well-understood. However, a number of changes in the prothrombotic coagulation factors have been reported in COVID-19, including elevated factor VIII, elevated fibrinogen, and increased viscosity [7]. Furthermore, there is evidence that the SARS-CoV-2 virus may invade the endothelial cells directly leading to cell injury and activating the coagulation cascade [8].

The spectrum of thromboembolic complications of COVID-19 is broad and ranges in severity from asymptomatic to organ dysfunction resulting in death [2]. Venous thromboembolism and pulmonary embolism (PE) are well-recognized complications of COVID-19, that were seen in up to 30% of patients in the intensive care unit according to initial reports [9]. Additionally, arterial thrombotic events such as stroke and myocardial infarction may occur, but they are less common than venous thrombosis in COVID-19 [10].

PE is a potentially life-threatening medical emergency. Early diagnosis and management defines the prognosis of PE as the mortality rate can reach up to 30% if the diagnosis of PE is missed or the management is delayed [11]. The clinical manifestations of PE are non-specific and have a significant overlap with those of COVID-19. Additionally, D-dimer levels are often elevated in patients with COVID-19, making it challenging to determine which patients require computed tomography pulmonary angiography (CT-PA) [12].

CT-PA is the diagnostic modality of choice for ruling out PE. Considering its widespread availability and high accuracy in making the diagnosis of PE, there is a low-threshold tendency for its overutilization. Hence, the positive rate of CT-PA for PE is often considered as an indicator of the appropriate use of the study. Limited studies have investigated the use of CT-PA in patients with COVID-19 in comparison with patients without COVID-19. Therefore, the aim of this study is to investigate the positive rate of CT-PA for PE among patients with COVID-19 in comparison to a control group.

## Materials and methods

Study design and setting

After obtaining approval from the ethics and research committee (IAU-IRB 2020-155), we conducted a retrospective study examining the diagnostic yield of CT-PA in patients with confirmed COVID-19 and compared it with patients without COVID-19. The study also aimed to identify the determinants of PE in patients with COVID-19. It was conducted at two major hospitals (Qatif Central Hospital and Dammam Central Hospital) in the Eastern Province of Saudi Arabia. In these institutions, the CT-PA scan can only be requested by board-certified physicians.

Study population

Eligible patients included all adult patients with COVID-19 confirmed by RT-PCR tests who underwent CT-PA for ruling out PE. Additionally, a similar number of patients without COVID-19 who underwent CT-PA were chosen randomly to be the control group. The hospital information system was utilized to identify all patients meeting the eligibility criteria who presented from June 2020 to June 2021. These included a total of 316 patients, including 158 patients with COVID-19.

Data collection and imaging technique

A structured data collection form was used to collect the data from the electronic health record. Data pertaining to demographic information such as date of birth, sex, and co-morbidities were obtained. Additionally, clinical information on presentation, including clinical symptoms and vital signs, was collected. D-dimer values for patients were obtained, if available. The Wells score of patients was calculated retrospectively using the available clinical data. The CT-PA scans were reviewed by board-certified radiologists to evaluate for the presence of filling defect suggestive of acute PE.

The scans were performed using the dual-source 128-slice scanner with the administration of 25 ml non-ionic contrast material with timed intravenous pump infusion followed by a 25-ml saline flush, after the test bolus. The injection rate was 4 ml/s and the scan was performed from the diaphragm to the lung apices.

Statistical analysis

The collected data was combined using Microsoft Excel (Microsoft, Redmond, WA, USA). Categorical data, presented as frequencies and percentages, were compared using the chi-square or Fischer exact tests. Continuous variables, presented as means and standard deviations, were compared using the independent t-test or analysis of variance test. The statement of significance was based on a significant level of alpha at 0.05. A multivariable regression analysis model was conducted to identify the predictors of PE among patients with COVID-19. All the analysis was conducted using IBM SPSS for Windows, version 25 (IBM Corp., Armonk, NY, USA).

## Results

Patient characteristics

The study included 316 patients, including 158 patients with COVID-19, who underwent CT-PA for ruling out PE. These included 200 (63.3%) male patients and 116 (36.7%) female patients. Most patients (72.2%) were aged below 50 years. Overall, 152 (48.1%) patients had a history of hypertension. Furthermore, 81 (25.6%) patients were smokers and 57 (18.0%) patients were obese. Only 40 (12.7%) patients had a previous history of pulmonary disease.

Regarding the clinical presentation of patients, dyspnea was the most frequent symptom seen in 225 (71.2%) patients. Fever was seen in 108 (34.2%) patients. Furthermore, 84 (26.5%) and 70 (22.2%) presented with chest pain and cough, respectively. Only 32 (10.1%) patients had an altered level of consciousness. In total, 218 (68.9%) patients had tachycardia and 179 (56.6%) had an oxygen saturation below 95%.

Over half (54.4%) of patients had elevated D-dimer levels. Leucocyte count was elevated in 204 (64.6%) patients. There were 184 (58.2%) and 160 (50.6%) patients having an elevated erythrocyte sedimentation rate and C-reactive protein level, respectively (Table 1).

**Table 1:** Characteristics of patients N, number of patients

Variable			N	%
Sociodemographic factors	Age (years)	18–34	94	29.7
		35–49	134	42.4
		50–65	59	18.7
		>65	29	9.2
	Gender	Male	200	63.3
		Female	116	36.7
	Comorbidities	Hypertension	152	48.1
		Diabetes mellitus	104	32.9
		Pulmonary disease	40	12.7
		Obesity	57	18.0
	Smokers		81	25.6
Clinical Features	Presenting symptoms	Dyspnea	225	71.2
		Chest pain	84	26.5
		Cough	70	22.2
		Fever	108	34.2
		Altered consciousness	32	10.1
	Tachycardia		218	68.9
	Decreased oxygen saturation		179	56.6
Laboratory findings	Elevated leucocyte count		204	64.6
	Elevated erythrocyte sedimentation rate		184	58.2
	Elevated C-reactive protein		160	50.6
	Elevated D-dimer		172	54.4

Comparison of the positive CT-PA rates

Seventy-six patients were found to have PE on the CT-PA scan, yielding a positive rate of 24.1%. However, there was a notable significant difference in the CT-PA positive rate according to the COVID-19 status. For example, only 13 (8.2%) patients with COVID-19 were found to have PE while 63 (39.9%) patients without COVID-19 had PE (P < 0.01).

There was no statistically significant between patients with COVID-19 and those without COVID-19 regarding their age and gender (P > 0.05). Furthermore, obesity was more prevalent among patients with COVID-19 (24.1% vs. 12.0%; P < 0.01). Similarly, diabetes mellitus was slightly more prevalent among patients with COVID-19 (36.1% vs. 29.7%), but the difference was not statistically significant (P = 0.23).

Regarding the clinical and laboratory findings, fever was more commonly seen in patients with COVID-19 (51.9% vs. 16.5%; P < 0.01). However, there was no significant difference in the prevalence of other presenting symptoms according to the COVID-19 status. Tachycardia was more frequent among patients without COVID-19 (87.3% vs. 50.6%; P < 0.01). In total, 138 (87.3%) patients with COVID-19 had elevated D-dimer levels compared with 34 (21.5%) patients without COVID-19 (P < 0.01). The difference between patients with COVID-19 and those without COVID-19 regarding the demographic, clinical, and laboratory findings is summarized in Table 2.

**Table 2:** Characteristics of patients according to the COVID-19 status N, number of patients; COVID-19, coronavirus disease 2019

Variable			COVID-19	Non-COVID-19	P value
			N (%)	N (%)	
Sociodemographic factors	Age (years)	18–34	54 (34.2)	40 (25.3)	0.07
		35–49	60 (38.0)	59 (37.3)	
		50–65	22 (13.9)	39 (24.7)	
		>65	22 (13.9)	20 (12.7)	
	Gender	Male	104 (65.8)	96 (60.8)	0.35
		Female	54 (34.2)	62 (39.2)	
	Comorbidities	Hypertension	72 (45.6)	87 (55.1)	0.09
		Diabetes mellitus	57 (36.1)	47 (29.7)	0.23
		Pulmonary disease	24 (15.2)	16 (10.1)	0.17
		Obesity	38 (24.1)	19 (12.0)	<0.01
	Smokers		44 (27.8)	37 (23.4)	0.37
Clinical features	Presenting symptoms	Dyspnea	100 (63.3)	115 (72.8)	0.07
		Chest pain	39 (24.7)	45 (28.5)	0.45
		Cough	38 (24.1)	32 (20.3)	0.42
		Fever	82 (51.9)	26 (16.5)	<0.01
		Altered consciousness	17 (10.8)	15 (9.5)	0.71
	Tachycardia		80 (50.6)	138 (87.3)	<0.01
	Decreased oxygen saturation		84 (53.2)	95 (60.1)	0.21
Laboratory findings	Elevated leucocyte count		92 (58.2)	102 (64.6)	0.25
	Elevated erythrocyte sedimentation rate		96 (60.8)	88 (55.7)	0.36
	Elevated C-reactive protein		82 (51.9)	78 (49.4)	0.65
	Elevated D-dimer		138 (87.3)	34 (21.5)	<0.01

Multivariable analysis of factors associated with PE among COVID-19 patients

A multivariable binary logistic regression analysis model was conducted to identify the independent factors associated with PE among patients with COVID-19. The model revealed that the smoking status (odds ratio [OR] = 1.94; 95% confidence interval [CI]: 1.4-3.8) and obesity (OR = 4.1; 95% CI: 1.5-8.9) were independent predictors of PE. However, the elevated D-dimer level was not significantly associated with PE among patients with COVID-19 (OR = 0.7; 95% CI: 0.4-1.8).

## Discussion

The study aimed to investigate the positive rate of CT-PA for PE in patients with COVID-19 and to identify the factors that serve as independent predictors of PE in such patients. The findings showed a significantly lower positive rate of CT-PA for PE among patients with COVID-19. Since coagulopathy became a well-recognized complication of COVID-19, the lower positive rate of CT-PA in COVID-19 patients in our study may suggest the overutilization of CT-PA.

It is interesting to note that despite the lower positive rate for PE among patients with COVID-19, the elevated D-dimer levels were more common among patients with COVID-19. In keeping with the shared clinical features between severe COVID-19 pneumonia and PE, the elevated D-dimer level is likely a contributor to the overutilization of CT-PA for ruling out PE in such patients. Studies found that COVID-19 causes inflammation with endothelial injury resulting in elevated D-dimer levels [12]. Hence, D-dimer testing is insufficient to be a standalone test for the diagnosis of PE. Accordingly, some researchers suggested the use of different cut-off values for D-dimer in patients with COVID-19 [13].

The low positive rate of CT-PA for PE in the present study is consistent with previous studies. For example, Birk et al. conducted a retrospective study including 285 consecutive patients with suspected COVID-19 who underwent CT-PA on a triage pathway [14]. Interestingly, they found that only one patient out of 48 patients with COVID-19 had PE compared with 25 patients out of 215 patients in the control group, suggesting that the prevalence of PE was lower in patients with COVID-19.

The study found that the smoking history is an independent factor associated with PE in patients with COVID-19. This is in line with previous literature which showed that current and former smokers are at higher risk of developing venous thromboembolism compared with non-smokers [15]. Therefore, interventional strategies aiming at increasing the awareness of the complications of COVID-19 among smokers are warranted.

To the best of our knowledge, this is the first study in Saudi Arabia to investigate the utilization of CT-PA in patients with COVID-19. However, the study has certain limitations. It is a retrospective study that may be limited by inaccurate or missing data about the clinical manifestations found in the electronic health records. Additionally, it is a two-center study and the results of this study may not be generalizable in all patients of COVID-19 due to variations in the practice and protocol of requesting medical imaging. Further studies are needed to confirm our findings.

## Conclusions

This study suggests the probable overutilization of the CT-PA scans in patients with COVID-19 as indicated by the significantly lower CT-PA positive rate for PE among these patients. The significantly higher proportion of elevated D-dimer values above the normal reference range in these patients is a possible contributor. Hence, this finding should prompt physicians to consider a higher cut-off value for D-dimer in patients with COVID-19. Furthermore, it is essential to keep in mind that patients with COVID-19 who are smokers were found to be at higher risk of PE. The present study provides valuable information on the potential hazards of smoking among COVID-19 patients, and such information can be used to raise community awareness.
